# Effect Observation on Modified Zishen Tongguan Decoction Combined with Acupuncture in Treatment of Urinary Retention after Cervical Cancer Surgery and Its Influence on the Incidence of Adverse Reactions

**DOI:** 10.1155/2021/7338276

**Published:** 2021-10-13

**Authors:** Shujuan Wang, Min Wang, Hongbin Zhang

**Affiliations:** ^1^Traditional Chinese Medicine Dispensing Room, Jinan Municipal Hospital of Traditional Chinese Medicine, Jinan 250012, Shandong Province, China; ^2^Department of Accupuncture, People's Hospital of Shizhong District of Jinan, Jinan 250024, Shandong Province, China

## Abstract

**Objective:**

To explore the effect observation on modified Zishen Tongguan decoction combined with acupuncture in the treatment of urinary retention after cervical cancer surgery and its influence on the incidence of adverse reactions.

**Methods:**

The clinical data of 84 patients suffered from urinary retention after radical resection of cervical cancer (December 2018–December 2019) in the oncology department of Jinan Municipal Hospital of Traditional Chinese Medicine were selected for retrospective analysis. According to the order of admission, they were divided into group A (*n* = 42), treated with conventional therapy, modified Zishen Tongguan decoction, and acupuncture, and group B (*n* = 42), treated with conventional therapy. The clinical efficacy of the two groups was observed, the urination function indexes after therapy were recorded, and the clinical efficacy and incidence of adverse reactions were analyzed.

**Results:**

After therapy, compared with group B, the average urinary flow rate, maximum urinary flow rate, bladder compliance (BC) level value, and the number of patients with good recovery of bladder function of group A were obviously higher (*P* < 0.05), and the urination time and detrusor pressure were obviously lower (*P* < 0.001). There was no significant difference in the average scoring of overactive bladder syndrome score (OABSS) between the two groups at 7 days of therapy (*p* > 0.05). The average OABSS of group A at 14 days of therapy was obviously lower than that of group B (*P* < 0.001). Compared with group B, the total clinical effective rate of group A was obviously higher (*P* < 0.05), while the total incidence of adverse reactions was obviously lower (*P* < 0.05).

**Conclusion:**

Modified Zishen Tongguan decoction combined with acupuncture is a reliable method to treat urinary retention after cervical cancer surgery, which greatly improves the urination function of patients, as well as the clinical efficacy. Further research will help create a better solution for patients with urinary retention after cervical cancer surgery.

## 1. Introduction

Cervical cancer is the primary malignant tumor of cervix, ranking first among women's malignant tumors in our country, with clinical manifestations of vaginal bleeding, swelling and pain of lower limbs, and unpleasant smell [1, 2]. Surgery is a common method to treat cervical cancer, but it affects a wide range of lesions and easily damages ligamentum and nerve fibers. Because of the long recovery time of bladder contraction after surgery, the incidence of urinary retention is very high. The symptom is that the urine in the bladder is filled to capacity and cannot discharge by itself, which is a common complication after cervical cancer surgery [3–5]. Urinary retention can cause urinary tract infection, resulting in dysuria. In addition, because the bladder cannot be emptied, bacterial infection is easy to occur and cystitis is caused. Currently, indwelling urinary catheter is mostly adopted in the clinic as a routine treatment method [6], which, although can alleviate the symptoms to a certain extent, has poor treatment effect due to the fact that long indwelling period can easily cause infection. Therefore, an effective treatment program for urinary retention after cervical cancer surgery is urgently needed. Some scholars have pointed out in their research [7] that the addition of traditional Chinese medicine (TCM) treatment on the base of conventional therapy such as urinary catheterization has significant effect, and the use of TCM to treat urinary retention has received widespread attention. TCM believes that the patients' vitality is badly sapped after surgery, their lung, spleen, and kidney are weak, and their waterways cannot be regulated, causing difficulty in urination [8]. Therefore, the treatment should be based on tonifying the kidney and qi and dissipating heat and stasis. Zishen Tongguan decoction has the effect of promoting blood circulation to remove blood stasis, tonifying the kidney, and inducing diuresis for treating stranguria, which can improve the urination function after surgery and accelerate rehabilitation of patients. Previous studies have shown that acupuncture can promote the voluntary movement of bladder to reduce the urinary dysfunction [9]. However, there are few reports about the combination of TCM and acupuncture in treating urinary retention after cervical cancer surgery. This study aims to provide more accurate data for the studies of Zishen Tongguan decoction combined with acupuncture in the treatment of urinary retention after cervical cancer surgery and provide some clinical reference.

## 2. Materials and Methods

### 2.1. General Data

The clinical data of 84 patients suffered from urinary retention after radical resection of cervical cancer (December 2018–December 2019) in the oncology department of Jinan Municipal Hospital of Traditional Chinese Medicine were selected for retrospective analysis. According to the order of admission, they were divided into group A (*n* = 42) and group B (*n* = 42). See Figure 1 for details.

### 2.2. Inclusion and Exclusion Criteria

The inclusion criteria were as follows: (1) all the enrolled patients met the diagnostic criteria for cervical cancer of *Guidelines for Diagnosis and Treatment of Cervical Cancer (4*^*th*^*edition)* [10] and were diagnosed by histopathology, and the clinical manifestations included contact bleeding, abnormal vaginal bleeding, abnormal vaginal discharge, and urgency of micturition; (2) all patients underwent radical resection of cervical cancer; (3) the patients suffered from postoperative urinary retention, and their residual urine volume was >100 ml; (4) the patients were diagnosed with urinary retention by ultrasonography and reproductive system examination; and (5) the patients were conscious, and their clinical data were complete.

The exclusion criteria were as follows: (1) the patients with urinary calculus; (2) the patients with liver and kidney dysfunction and immune disease; (3) the patients with other severe postoperative complications such as pelvic infection, lymphocyst, postoperative bleeding, and urethrovaginal fistula; (4) the patients with bladder dysfunction; and (5) the patients who were allergic to the medicine in this study.

The study was approved by the ethics committee of Jinan Municipal Hospital of Traditional Chinese Medicine, and all the patients and their families knew the study and signed the informed consent.

### 2.3. Methods

After surgical treatments including extensive hysterectomy and laparoscopic pelvic lymph node resection, all patients had urinary retention after surgery, received indwelling urethral catheter, and orally took the prazosin hydrochloride tablets (manufactured by Changzhou Pharmaceutical Factory Co., Ltd., NMPA approval no. H32023906; specification: 1 mg × 100 tablets/bottle). Meanwhile, physical stimulation, such as hot compress, massage of bladder area, and listening to the sound of water flow, was applied to patients. The urine bag was changed and perineum was disinfected once a day [11].

Patients in group A were additionally treated with modified Zishen Tongguan decoction combined with acupuncture. Zishen Tongguan decoction included, respectively, 20 g of Chinese yam, Cortex Phellodendri, Rhizoma Anemarrhenae, cowherb seed, and Poria; 10 g of Rhizoma Alismatis, lycopodii herb, Cortex Moutan Radicis, *Polyporus umbellatus*, and *Cornus officinalis*; 50 g of Radix Astragali; 15 g of Fructus aurantii, Prepared Radix Rehmanniae, Peach Kernel, and *Achyranthes* root; 8 g of Radix Aconiti Carmichaeli and Cortex Cinnamomi; 12 g of Rhizoma Sparganii and Rhizoma Curcumae; and 6 g of liquorice root. The patients were administrated with the decoction for 50 ml each time and 3 times a day (the decoction was decocted with water). If the patients were accompanied by red complexion, irritability, red urine, constipation, and yellow tongue with red coating, the illness was diagnosed as toxic heat. 10 g of Hemp Fruit and mirabilite, respectively, should be added. If the patients had heaviness sensation in the limbs and head, recessive fever, bitter taste, yellow urine, little urinary volume, chest fullness, and red tongue with yellow coating, the illness was diagnosed as internal damp-heat. 20 g of capillary *Artemisia* and 30 g of gentian should be added. If the patients were accompanied by tiredness, abdominal distension, epigastric discomfort, diarrhea, and pale tongue with white coating, the illness was diagnosed as stagnancy of cold-dampness. 6 g of Manchurian Wildginger, 15 g of parasitic *Loranthus*, and 10 g of Chinese teasel root should be added. If the patients had feverish sensation over the palm and sole, pale complexion, tiredness, and red tongue with little coating, the illness was diagnosed as deficiency of qi and yin. 15 g of Radix Scrophulariae and 20 g of Polygonatum odoratum, *Ophiopogon japonicus*, Radix Rehmanniae, and *Dendrobium* should be added.

#### 2.3.1. Acupuncture Therapy

The patients received acupuncture therapy from the 4^th^ day after surgery. The lateral position was taken. Yinlingquan, Qihai, Guanyuan, Zusanli, Baihui, bilateral Sanyinjiao, and bladder meridian acupoints were selected for acupuncture. After routine disinfection, twirling-reinforcing- and uniform reinforcing-reducing needling methods were used. The retaining needle time for the above acupoints was 30 min. The acupuncture was conducted once a day. Both groups were treated for 21 consecutive days, and the therapeutic outcome was observed [12, 13].

### 2.4. Observation Indexes

An intelligent urinary flow rate detector (manufacturer: Beijing Zhongxi Huada Technology Co., Ltd.; model: CN202M272181) was used to detect the average urinary flow rate, maximum urinary flow rate, and urination time of the two groups after therapy. Urodynamic analyzer (manufacturer: Beijing Haifuda Technology Co., Ltd.; model: ZN999-Nidoc970A) was used to detect detrusor pressure and bladder compliance (BC) level value.

Residual urine volume ≤100 ml indicated good recovery of bladder function. The number of patients with good recovery of bladder function in both groups after therapy was evaluated.

Urination situation at 7 days and 14 days of therapy of the two groups was evaluated according to overactive bladder syndrome score (OABSS) [14]. The scale included urination frequency during daytime, urination frequency at night, urinary urgency, and urge urinary incontinence, with the total score of 15 points. The higher the score, the more severe the overactive bladder syndrome.

Evaluation of clinical symptoms: (1) if the urinary retention disappeared, urination was smooth, and residual urine volume was not more than 50 ml, it was cured. If the urinary retention basically disappeared, urination was a little blocked, and residual urine volume was 51–100 ml, it was markedly effective. If the urinary retention was reduced, urination lasted longer, there was painful and uncomfortable urination, and residual urine volume was 51–100 ml, it was effective. If the patients could not urinate by themselves, it was invalid.

The incidence of adverse reactions of the two groups was recorded, including rash, salivation, urinary system infection, and nausea and vomiting.

### 2.5. Statistical Methods

The data processing software selected in this study was SPSS21.0, and the selected drawing software was GraphPad Prism 7 (GraphPad Software, San Diego, USA). The count data were tested by the *X*^2^ test and described by (*n* (%)). The measurement data were tested by the *t* test and described by mean ± SD. *P* < 0.05 indicated that the difference had statistical significance.

## 3. Results

### 3.1. Comparison of the Baseline Data

There was no significant difference in baseline data including mean age, BMI, disease types, and clinical stages between the two groups (*P* > 0.05), as shown in Table 1.

### 3.2. Comparison of the Urination Situation after Therapy

After therapy, compared with group B, the average urinary flow rate and maximum urinary flow rate of group A were obviously higher, while the urination time and detrusor pressure were obviously lower (*P* < 0.001). See details in Table 2.

### 3.3. Comparison of the Number of Patients with Good Recovery of Bladder Function and BC Level Values after Therapy

After therapy, the BC level value and the number of patients with good recovery of bladder function of group A were obviously higher compared with group B (*P* < 0.05), as shown in Figure 2.

### 3.4. Comparison of the OABSS Scores at 7 and 14 Days of Therapy

There was no significant difference in the average OABSS scores between the two groups at 7 days of therapy (*P* > 0.05). The average OABSS score of group A was obviously lower compared with group B at 14 days of therapy (*P* < 0.001). See details in Figure 3.

### 3.5. Comparison of the Clinical Efficacy

The total clinical effective rate of group A was obviously higher compared with group B (*P* < 0.05), as shown in Table 3.

### 3.6. Comparison of the Incidence of Adverse Reactions

The total incidence of adverse reactions of group A was obviously lower compared with group B (*P* < 0.05), as shown in Table 4.

## 4. Discussion

Cervical cancer is one of the most common diseases affecting women's health, and the continuous infection with high-risk human papillomavirus (HPV) is the most important pathogenic factor in the occurrence and development of it [15, 16]. Surgical resection is often used clinically, which has better therapeutic effect. However, because of the large trauma area of the surgery and intraoperative free ureter lower end, the peripheral nerve of the bladder may be removed when upper pushing the bladder, thereby causing postoperative bladder dysfunction and then the occurrence of urinary retention [17]. In addition, because of the mental stress caused by postoperative pain, being unaccustomed to urinating in bed, and urinary tract infection caused by urinary catheter insertion, the possibility of urinary retention will also increase, which may result in pyelitis, obstruction of the ureter, ureteral fistula, and other complications, affecting the postoperative recovery. At present, indwelling urinary catheter combined with Western medicine is often used as a conventional therapy. Although it can relieve clinical symptoms to a certain extent, urinary tract infection may be caused by long-term indwelling catheter, with limited efficacy [18].

It has been reported [19] that the implementation of TCM treatment in patients with urinary retention after mixed hemorrhoid surgery can stimulate the bladder and induce diuresis. TCM believes that urinary retention belongs to the category of uroschesis. Kidney qi deficiency, lack of vitality after surgery, and unregulated waterways can result in inability to urinate normally and retention of the bladder. Therefore, the therapy should be based on tonifying the kidney and qi, removing blood stasis, and alleviating water retention [20]. In this study, the therapeutic effect of modified Zishen Tongguan decoction combined with acupuncture on urinary retention after cervical cancer surgery was observed. Modern pharmacological studies have shown [21] that Radix Astragali has the effect of replenishing vitality, antiaging, enhancing immunity, and inducing diuresis. Rhizoma Anemarrhenae can nourish the kidney and yin, clear heat, and drain fire, which has antibacterial and antitumor effect. Rhizoma Alismatis is cold-natured, which can remove dampness and promote diuresis after entering the kidney and bladder meridian. Polyporus umbellatus plays a role of inducing diuresis and curing edema. Polyporus polysaccharide injection was subcutaneously injected to rats by some scholars [22], and significant increase of urine volume was found in the rats. The combined use of the above herbal medicine can make patients' kidney-qi sufficient, bladder gasification normal, and urination smooth. Acupuncture takes patients' acupoints as the point of penetration, which can treat disease of internal organs. Guanyuan, Yinlingquan, Zusanli, etc., are selected for regulating the bladder and assisting in gasification. Yilingquan is selected for promoting blood circulation to remove blood stasis and clearing heat and dampness. Acupuncture on the above points has the effect of dredging meridians, promoting qi to induce diuresis, solid off, and addendum [23].

This study showed that compared with group B, the average urinary flow rate and maximum urinary flow rate of group A after therapy were obviously higher, while the urination time and detrusor pressure were obviously lower (*P* < 0.001). It is speculated that Zishen Tongguan decoction combined with acupuncture can affect neuronal activity, promote the contraction of sphincter and detrusor, and enhance urinary function. BC refers to the ability to maintain constant pressure or slightly increase pressure, which is the tolerance of the bladder to the increased fluid [24]. This study showed that the BC level value of group A after therapy was obviously higher compared with group B (*P* < 0.001). It is speculated that acupuncture plays a role during the treatment, which can regulate yin and yang of viscera and promote the functional recovery of bladder smooth muscle through stimulating acupoints. Cowherb seed and Rhizoma Alismatis included in the decoction can stimulate nerve conduction, increase the blood perfusion of the local vessels of the bladder detrusor, and promote the recovery of tissue, which has been confirmed in the study of Nardone et al. [25]. The study also showed that the incidence of adverse reactions of group A was obviously lower compared with group B (*P* < 0.05), indicating that Chinese herbal decoction combined with acupuncture had high safety and could improve the therapeutic effect. Deficiencies of this study were as follows. The clinical trial lasted for 3 weeks due to the limitation of the research cycle, and the long-term efficacy of the patients after therapy could not be completely followed up. Therefore, the experimental design scheme needed to be improved. There was a lack of research on emotional changes and quality of life of patients. It is hoped that the impact on the life and mental health of such patients could be evaluated in future studies.

In summary, the modified Zishen Tongguan decoction combined with acupuncture can significantly improve the therapeutic effect, bladder compliance, and urinary function in patients with urinary retention after cervical cancer surgery. Therefore, the combined use of modified Zishen Tongguan decoction and acupuncture has high clinical value.

## Figures and Tables

**Figure 1:** Route of experimental technique.

**Figure 2:** Comparison of the number of patients with good recovery of bladder function and BC level values after therapy (*n* (%), mean ± SD). (a) Comparison of BC level values between the two groups after therapy. The horizontal axis represents group *A* and group *B*, and the vertical axis represents BC level value (ml/H_2_O). After therapy, the BC level values in group *A* and group *B* were 64.35 ± 8.34 ml/H_2_O and 56.23 ± 8.46 ml/H_2_O, respectively. ^*∗*^There was a significant difference in BC level values between the two groups after therapy (*t* = 4.430, *P* < 0.001). (b) Comparison of the number of patients with good recovery of bladder function between the two groups after therapy. The horizontal axis represents group A and group B, and the vertical axis represents the number of patients with good recovery of bladder function (*n* (%)). After therapy, the number of patients with good recovery of bladder function in group A and group B were 39 (92.86%) and 32 (76.19%), respectively. ^*∗∗*^There was a significant difference in the number of patients with good recovery of bladder function between the two groups after therapy (*X*^2^ = 4.459, *P* < 0.05).

**Figure 3:** Comparison of OABSS scores at 7 d and 14 d of therapy (mean ± SD, *n* = 42). (a) Comparison of OABSS scores between the two groups at 7 d of therapy. The average OABSS scores of group A and group B at 7 d of therapy were 9.17 ± 1.72 points and 10.40 ± 1.67 points, respectively. (b) Comparison of OABSS scores between the two groups at 14 d of therapy. The average OABSS scores of group A and group B at 14 d of therapy were 5.58 ± 1.50 points and 7.98 ± 1.60 points, respectively. The horizontal axis represents group A and group B, and the vertical axis represents OABSS score (points). ^*∗*^There was a significant difference in average OABSS scores between the two groups at 14 d of therapy (*t* = 7.092, *P* < 0.001).

**Table 1:** Comparison of baseline data (*n* = 42).

Items	Group A	Group B	*X* ^2^/*t*	*P*
Mean age (mean ± SD, years old)	42.18 ± 3.46	42.23 ± 3.42	0.067	0.947
BMI (mean ± SD, kg/m^2^)	21.82 ± 1.03	21.76 ± 1.06	0.263	0.793
*Disease types (n (%))*				
Squamous cell carcinoma	28 (66.67%)	25 (59.52%)	0.460	0.498
Adenocarcinoma	7 (16.67%)	9 (21.43%)	0.309	0.578
Squamous cell carcinoma and adenocarcinoma	5 (11.90%)	7 (16.67%)	0.389	0.533
Small cell carcinoma	2 (4.76%)	1 (2.38%)	0.346	0.557

*Clinical stages (n (%))*				
Stage IB2	13 (30.95%)	11 (26.19%)	0.233	0.629
Stage IIA1	17 (40.48%)	19 (45.24%)	0.194	0.659
Stage IIA2	9 (21.43%)	11 (26.19%)	0.263	0.608
Stage IIB1	3 (7.14%)	1 (2.38%)	1.050	0.306
Surgery time (mean ± SD, min)	155.48 ± 29.18	155.36 ± 30.19	0.019	0.985
Bladder urinary retention (mean ± SD, ml)	473.46 ± 36.74	475.25 ± 35.62	0.227	0.821
*Physical work (n (%))*			0.441	0.507
Yes	26 (61.90%)	23 (54.76%)		
No	16 (38.10%)	19 (45.24%)		
*Surgical approaches (n (%))*			0.202	0.653
Laparoscopic surgery	27 (64.29%)	25 (59.52%)		
Laparotomy	15 (35.71%)	17 (40.48%)		
*Marital status (n (%))*				
Married	6 (14.29%)	8 (19.05%)	0.343	0.558
Unmarried	34 (80.95%)	31 (73.81%)	0.612	0.434
Divorced	2 (4.76%)	3 (7.14%)	0.213	0.645

*Residence (n (%))*			0.778	0.378
Cities and towns	16 (38.10%)	20 (47.62%)		
Countryside	26 (61.90%)	22 (52.38%)		
*Education level (n (%))*				
College and above	8 (19.05%)	7 (16.67%)	0.081	0.776
High school	25 (59.52%)	21 (50.00%)	0.769	0.381
Middle school and below	9 (21.43%)	14 (33.33%)	1.497	0.221

**Table 2:** Comparison of urination situation after therapy (mean ± SD, *n* = 42).

Items	Average urinary flow rate (cm/s)	Maximum urinary flow rate (cm/s)	Urination time (s)	Detrusor pressure (cm·H_2_O)
Group A	8.32 ± 1.36	16.27 ± 2.27	34.18 ± 4.63	22.17 ± 3.18
Group B	6.27 ± 1.42	12.96 ± 2.31	41.26 ± 4.73	28.12 ± 3.21
*t*	6.757	6.623	6.932	8.534
*P*	＜0.001	＜0.001	＜0.001	＜0.001

**Table 3:** Comparison of clinical efficacy (*n* (%)).

Items	*n*	Cured	Markedly effective	Effective	Invalid	Total clinical effective rate
Group A	42	23 (54.76)	11 (26.19)	6 (14.29)	2 (4.76)	95.24% (40/42)
Group B	42	17 (40.48)	9 (21.43)	8 (19.05)	8 (19.05)	80.95% (34/42)
*X* ^2^						4.087
*P*						<0.05

**Table 4:** Comparison of incidence of adverse reactions (*n* (%)).

Items	*n*	Rash	Salivation	Urinary tract infection	Nausea and vomiting	Total incidence
Group A	42	1 (2.38)	0 (0.00)	0 (0.00)	2 (4.76)	7.14% (3/42)
Group B	42	2 (4.76)	1 (2.38)	4 (9.52)	3 (7.14)	23.81% (10/42)
*X* ^2^						4.459
*P*						<0.05

## Data Availability

The data used to support the findings of this study are available on reasonable request from the corresponding author.
